# An analysis of machine learning risk factors and risk parity portfolio optimization

This article has been retracted.

**DOI:** 10.1371/journal.pone.0272521

**Published:** 2022-09-26

**Authors:** Liyun Wu, Muneeb Ahmad, Salman Ali Qureshi, Kashif Raza, Yousaf Ali Khan

**Affiliations:** 1 School of Trade and Economics, Shanghai Urban Construction Vocational College, Shanghai, PR China; 2 School of Finance, Jiangxi University of Finance and Economics, Nanchang, Jiangxi, China; 3 Department of Business Administration, Allama Iqbal Open University, Islamabad, Pakistan; 4 Division of Management and Administrative Sciences, UE Business School, University of Education Lahore, Lahore, Pakistan; 5 Department of Mathematics and Statistics, Hazara University Mansehra, Mansehra, Pakistan; Hanyang University, REPUBLIC OF KOREA

## Abstract

Many academics and experts focus on portfolio optimization and risk budgeting as a topic of study. Streamlining a portfolio using machine learning methods and elements is examined, as well as a strategy for portfolio expansion that relies on the decay of a portfolio’s risk into risk factor commitments. There is a more vulnerable relationship between commonly used trademarked portfolios and neural organizations based on variables than famous dimensionality decrease strategies, as we have found. Machine learning methods also generate covariance and portfolio weight structures that are more difficult to assess. The least change portfolios outperform simpler benchmarks in minimizing risk. During periods of high instability, risk-adjusted returns are present, and these effects are amplified for investors with greater sensitivity to chance changes in returns R.

## 1. Introduction

Numerous academic and professional inquiries are focused on portfolio development and risk management. Breaking down the portfolio’s risk into peril figure obligations provides an approach for portfolio development in this study. The study evaluates latent components’ features and advantages of machine learning dimensionality reduction for asset appropriation. Covariance grids, which are utilized to build least-distinct portfolios, focus on the investigation. PLS can be used to transform an enormous amount of information about the expected returns from an assortment of business variables into a few composite parts that predict the cross-segmentation of anticipated stock returns [1]. Components with a low degree of series variation identify benefits in the cross-section of benefits using a PCA [2]. Auto-encoders, a type of neural engineering used to reduce dimensionality, are also examined in this study. The framework the study uses to overcome any barrier between Machine learning and cash is the source of our responsibilities. Latent components, like component-based covariance grids, are examined for their impact on the formulation and implementation of least-contrast portfolios. These portfolios and extended Sharpe degrees for the US respect market utilize a variety of part-based covariance frameworks [3]. The study aims to analyze data related to machine learning risk factors and risk parity portfolio optimization and determine that the minimum variance and maximum diversification are most sensitive to covariance misspecification. The study constructs least-change portfolios that focus on a certain portion and covariance highlight based on data from more than half-century US company portfolios. The study also aims to determine the impact of the various time horizons for rebalancing and how the portfolios compare to a market equally weighted portfolio. The results suggest that machine learning increases the value of assets based on parts, as proved by the findings of [4], and machine learning can enhance factor-based portfolio expansion when execution is approximated. Machine learning can increase factor-assembled portfolios by 3.2%, 1.55%, and 2.09% over the comparative weighted portfolio. An equally weighted portfolio would be valued between 3.04% and 5.2% higher by financial allies with moderate risk attitudes who apply machine learning aspects. PCA techniques regularly beat the same weighted benchmark, and auto-encoders with more mystery layers and directed approaches may be blamed for poor portfolio performance following the results of PLS and PCA [5]. It is concluded that using an equally-weighted risk factor responsibilities technique on the portfolio’s assets is comparable to a risk arrangement strategy with a specific risk monetary arrangement profile. A discussion follows on how to build a more robust version of risk parity optimization by integrating uncertainty structures to market parameters in the risk parity optimization model. A regime-switching risk parity portfolio based on the Fama-French three-factor model is tested in the study.

The structure of the paper is as follows the outline for this document: Section 2 of the study report demonstrates the methodology, data gathering methods, and research design. The machine learning techniques of latent Factors are matched with risk budgeting and machine learning methods of reaching for a concentration index in Section 3. Section 4 concludes with our portfolio development techniques’ future proposals and practical implementations.

## 2. Literature review

[6] used the elastic net to investigate the predictability of foreign stock returns, and [7] gave a complete comparison of machine learning approaches for the equities, bond, and hedge fund markets. More recently [8], have demonstrated the benefits of factor optimization by machine learning. Rather than using auto-encoders [9], employed a five-factor model. An asset-budgeting strategy would be risk-budgeting on the portfolio’s assets with a defined risk budget. Instrumental PCA (IPCA) is proposed by [10], where variables are latent, and the time-varying loadings depend on features. These findings suggest that a limited number of factors can better describe the average returns of the cross-section than other leading factor models do. After then [11], used machine learning to further the study without relying on IPCA’s linearity assumption. Additionally, there are PLS-related articles published in the financial literature. Using PLS [1], creates a model for predicting the cross-section of predicted stock returns based on data gathered from a wide number of business attributes. [2] presented risk premia PCA to find variables with minimal time-series fluctuation, which finds factors beneficial in a cross-section of returns. [12] discovered that a stochastic discount factor with a few main components, utilizing Bayesian shrinkage to choose a subset of attributes, gives strong out-of-sample explanatory power for average returns from a short sample. Among practitioners and academics alike, the mean-variance paradigm for portfolio optimization is still a favorite because elegant and has strong theoretical foundations [13]. It benefits from adopting risk factors to account for the key nutrients in our investment portfolios appropriately. The factor-based paradigm makes understanding and optimizing portfolios easier [14]. Under a set of equally likely asset return scenarios [15], offers a convex formulation of risk parity using CVaR and incorporates the downside risk measures into the proposed methods. Risk planning focuses on the portfolio’s risk expansion by assigning objective risk commitments to each portion. [16] introduced the concept of risk equality in that all risk obligations in a portfolio are equalized. Bridgewater Partners sent out the major danger reserve for equality in 1996, and it’s still there today and employed as a primary speculative strategy for businesses [17]. However, their approach is seen as subjective compared to current providers of risk-equivalent procedures [18]. Financiers and financial organizations have been motivated to support machine learning-supported trading procedures by significant breakthroughs in machine learning and deep learning processes [19]. Machine Learning methodologies and concepts used in the building of portfolios. Portfolio improvement is addressed by [20], use the machine learning and deep learning methods have been preferred by researchers across different disciplines for providing solutions to their problems. [21] use a Rope technique to choose quality attributes in a parametric portfolio problem. The base change method is one of several popular risk-based portfolio distribution approaches that only rely on covariance estimations. In a financial plan based on [22], with the highest expansion [23], A similar level of risk commitment is demonstrated by [24]. [25] provide an alternative, more computationally productive approach to the problem of danger equality and investigate scenarios in which the arrangement space may not be arched due to various financial plan needs [26]. Comparatively, the experimental presentation of risk equality portfolios is measured compared to other regular resource allocation techniques, such as mean-change improvement. [27] proposed an elective approach to risk equality that an alternative danger equality portfolio is produced by deconstructing a portfolio based only on its concealed danger measurements using head-part analysis (PCA). [28] looked at ways that machine learning advancements are used to address the forced quadratic programming problem from its root. According to [29], static portfolio advancement is defined as the prize, risk, and distinct conditions for optimal portfolios. The problem of risk management portfolios has gained traction among academics, and a growing body of work focuses on the features’ theoretical and computational aspects. According to [30] the portfolio risk equality model was conducted using a curve under long-justified spending plan requirements at the commencement of an extensive investigation. According to [31] concentrates on a more general form of risk-planning portfolios and calculated that the returns on a risk equality portfolio might be modest for certain investors, and [32] presents casual risk equality by combining the objective return imperatives. [33] provide an even more summarized version of equal risk portfolios with projected return constraints. Neuronal networks with differentiable enhancement layers that encode risk planning were created by [34] and determined that the issue of improvement is regarded as a differentiable layer in the company, where limits are learned via back-spreading. [26] found that academics and specialists are interested in a wide range of risk management techniques, including weighted and vacillating and most extensive portfolio weighted peril duties [35]. Compared to portfolios using more commonly used covariance assessors, the least difference portfolios show fewer changes and greater Sharpe proportions. Using a sophisticated shrinkage assessor [36], considers that the approaches such as "similarly weighted," "least change," and "most differentiated" portfolios. Similarly, weighted" danger commitments, "risk planning," and "expanded danger equality procedures" have become popular among academics and experts alike [37] and provide rich and efficient methods for handling the improvement of enhanced portfolios. Mean Variation (MV) [38], has been widely regarded as grounds for current portfolio theory. [39] encouraged portfolio executives to use a minimum method to estimate risk as to the portfolio’s base return over all previous perceptual time frames. For portfolio progression models based on CVaR [40], assures that CVaR manages common setbacks at a specific degree of certainty and computational capacity. [41] first introduced the disadvantage risk and is presently the most widely used risk assessment tool. Contingent worth in risk is one of the most important rational risk measures [42]. Because portfolio managers increasingly employ the mean-CVaR model [43] to build research portfolios for data analysis, the study utilized this approach. Hence CVarR is the ideal methodology for simplifying a problem [44]. Most minor capacity portfolios and element-based covariance connections are affected by the suggested inactive sections, a clear representation of the approaches for reducing CVaR [45]. When deciding on long-short portfolio allocations, [46] identified a constantly rising improvement in the use of execution destinations and risk metrics, including the unpredictability of VaR and CVaV. As opposed to MVO portfolios [47], says assessment mistakes less influence risk equality portfolios.

## 3. Research methodology

### 3.1 Data collection and analysis techniques

The research has collected the USA firms’ portfolio data of 49 industry-based portfolios. In contrast, the second has 21 assets, including 20 size-based portfolios, the S&P 500 from the website http://www.hedgeindex.com and the Kenneth R. French-Data Library website https://mba.tuck.dartmouth.edu provided monthly Net Asset Value (NAV) data for the global index. The data set of portfolios of all 49 companies outperformed the EW consignment in terms of standard deviation and Sharpe ratio from the Center for Research in Security Prices (CRSP), including monthly total individual stock returns from 1970 to 2020 (50 years data). Only stocks traded on the NYSE, AMEX, and NASDAQ databases are included. To analyse the data we have utilized MATLAB, function (*p = Portfolio(p*,*’AssetMean’*, *m*,*’AssetCovar’*,*C*) and R-studio functions(*model<optimal*.*portfolio(scenario*.*set);portfolio*.*weights(optimal*.*portfolio(scenario*.*set));portfolio*.*optimization-package;*harpe_ratio<-port_returns/port_risk).Microsoft’s *Excel* version-10 used 49 industry-based portfolios and another 21 resources, including 28 portfolios based on size and book-to-advertise (BM).

#### 3.1.1 Hypothesis development

**H**_**01**_: Machine learning methods lead to covariance and portfolio weight structures that deviate from simpler estimators.
**H**_**02**_: Auto encoder-derived minimum-variance portfolios beat simpler benchmarks regarding reducing risk.
**H**_**03**_: To solve the problem of portfolio allocation and the risk budgeting factor helps to develop a specific risk profile.
**H**_**04**_: Utilization of the mean absolute deviation (MAD) and conditional value at risk (CVaR) is a good effort to optimize the low and high-risk portfolios.

### 3.2 Research design

#### 3.2.1 Portfolio optimization with factor risk budgeting

One of the fascinating topics for many experts is coordinating plans for risk expenditures involving risk aspects. Research presented an alternate method for calculating the effective number of bets for risk budgeting and parity [37]. Keeping the amount of risk focused on each component to a minimum allows us to broaden our view of what constitutes "genuine" sources of risk. It can solve the portfolio designation problem by breaking the stake into its components.

#### 3.2.2 Matching the risk budgets

Risk budgeting is used as a portfolio allocation technique in which the allocation of risk is used to establish the portfolio’s weighted values. To create a risk-budgeting portfolio, each asset in the portfolio must contribute its fair share to meet the total budget. Building a risk budgeting portfolio with risk contributions that fit a set of specified risk budgets is aiming to do here {*a*_1_,…,*a*_*m*_}

$$SD(X_{i})=a_{j}\;S(y)$$ (1)

According to [48], the generic study problem may be expressed as a quadratic problem.


$${(x}^{*},{\hat{x}}^{*})=arg\;min\;\sum_{i=1}^{n}{\left(SD(X_{i})-a_{i}S(x,\tilde{x})\right)}^{2}$$

$$u.c\left\{ \begin{array}{c} 1^{T}D^{+}x+1^{T}{\tilde{D}}^{+}x=1\\ 0≼D^{+}x+{\tilde{D}}^{+}x≼1 \end{array}\right.$$ (2)

The first restriction that denotes inequalities among elements is a budget constraint, meaning that all of the portfolio’s assets are fully invested, but the second constraint prohibits short selling. If the objective function is equal to zero at the optimum, (1) there is a solution to the optimization issue; (2) it is also the matching problem. For a portfolio with a Sharpe Ratio of 1, the investor decides to invest in a leveraged long-short portfolio to meet the following constraints: Each asset I in the portfolio’s absolute contribution to total risk is assigned a risk budget of RB percent.


$$z_{i}.n_{i}\leq RB\%\;of\;\partial_{q},\;i=1,2,\ldots \ldots M$$ (3)

Wherever*n*_*i*_ is the not important expense to the risk of asset *i*, *z*_*i*_ is the weight of asset *i*, and ∂_*q*_ is the portfolio risk

$$\sum_{i=1}^{M}z_{i}=1$$ (4)

Unbounded inequality limits are put on certain assets reflecting the portfolio’s leverage

$$z_{i}>0\;or\;z_{i}\geq 0,\;i\neq j$$ (5)

—a limit placed on certain assets to create a leveraged long-short portfolio mix

$$b_{i}\geq z_{i}\geq -\alpha_{i}$$ (6)

Wherever (−*α*_*i*_, *b*_*i*_) free lower and upper limits −*α*_*i*_, *b*_*i*_ promoting an investor-friendly leveraged portfolio. The risk-budgeted portfolio is a leveraged long-short portfolio with three asset classes, each with particular limitations. Some high-yielding investments need leveraged investment (*z*_*i*_>0), additional high-yielding assets with leveraged investment (*w*_*j*_>0), and other unbound yet leveraged and long-short assets (*b*_*i*_≥*z*_*i*_≥ −*α*_*i*_). Let *Z*^+^, *Z*^*Spl*^, with *Z*^*Free*^ specify the three asset modules. The problem model is mathematically expressed as follows:

$$Max\;\left[\frac{\bar{q}.\bar{z}}{\sqrt{\bar{z}.U.\bar{z}}}\right]\;(maximize\;Sharpe\;Ratio)$$ (7)

Where $\bar{q}$ represents the *premia* (returns) of the assets in the portfolio, $\bar{z}$ the weights, and *U* the variance-covariance matrix of asset returns, $\bar{q}.\bar{z}$ is the expected portfolio return, $\partial_{q}=\sqrt{\bar{z}.U.\bar{z}}$ is the portfolio risk, and $\left[\frac{\bar{q}.\bar{z}}{\sqrt{\bar{z}.U.\bar{z}}}\right]$ is the Sharpe ratio of the portfolio, subject to the constraints,

$$RB\%\geq z_{i}.n_{i}\;of\;\partial_{q},\;i=1,2,\ldots ..,M\;(risk\;budgeting)$$ (8)

Where $\bar{n}=(n_{1},n_{2},\ldots .,n_{M})=\frac{\left(U.\bar{z}\right)}{\sqrt{\bar{z}.U.\bar{z}}}$ are the marginal contributions to risk, and *RB*% is the risk limit,

$$\sum_{i=1}^{M}z_{i}=1\;(Fully\;invested)$$ (9)

$$z_{j}^{+}>0\;(Financial\;leverage)$$ (10)

Where *Z*^+^ is the weights of selective positive premia assets *Z*^*sql*^,

$$z_{k}^{sql}\geq 0,j\neq k\;(optional\;inclusion\;of\;special\;leveraged\;assets)$$ (11)

Where $w_{k}^{sql}$ is the weight of some special assets, *W*^*sql*^, inclusion is optional if optimality requires but can be exploited to any amount if included

$$b_{i}\geq z_{i}^{Free}\geq -\alpha_{i}\;(Long‐short\;mix,\;promoting\;leveraging)$$ (12)

Where (−*α*_*i*_, *b*_*i*_) are free bounds for any *α*_*i*_, *b*_*i*_ acceptable to the investor for selective assets belonging to *Z*^*Free*^ and promoting a leveraged long-short portfolio. Equations (v-x) describe a single goal non-linear restricted fractional programming model that requires metaheuristic approaches to solve. The study applied the metaheuristic techniques and must use specific procedures that may require changing the original problem model.

#### 3.2.3 Sharpe ratio model

[49; 09] three-factor models are followed in this study, as well as their observable components, such macroeconomic indicators. A factor model for all asset returns *s*_*i*_ between j = 1, …, M assets, *t* = 1, …, *T* comments with *k* = 1, …, k experiential factors receive the equation:

$$s_{i}=\beta_{i}+\alpha_{i}X_{i}+\nu_{i}$$ (13)

where *α*_*i*_ = (*α*_*i*_,1, …, *α*_*i*_,k) are the issues’ time variation aspect loadings *X*_*t*_ = (*F*_*t*_,1, …, *F*_*t*_,k), *α*_*i*_ is the time-invariant interrupt, and is the time-invariant interrupt *v*_*i*_,*t* is the inaccuracy span for asset *i* at date *t*. As a result, OLS can estimate intercept and factor loadings using various factor representations and extract factors from latent variables. The principal component analysis is frequently utilized to reduce the dimensionality of latent components:

$$s_{i}=\beta_{i}+(Y_{t}Z)+\upsilon_{i},=\beta_{i}+\alpha_{i}X_{t}+\upsilon_{i},$$ (14)

Where Y_*t*_ = (y_1_, …, *x*_q_,_*t*_) is the *T*×q matrix of forecasters and Z = (z_1_, …, *z*_*k*_) is the q × k matrix of weights, with *K* "q. Each *z*_*k*_ is the vector of weights used to construct the *k*^th^ latent factor, *F*_*k*_; the *T*×k matrix of latent factors is given by x_*t*_ = Y_*t*_Z. The dimensionality of the data is decreased by translating the set of ***q*** predictors to a smaller number of ***k*** variables.

#### 3.2.4 PLS and PCA techniques

Incomplete least squares and head part inspection are two well-known techniques for reducing dimensionality. The factors may be modeled using the partial least squares (PLS) multivariate approach, and covariance between independent and dependent block scores is maximized by calculating these variables [50]. The indicators’ data *Y*_*t*_, whereas in PLS, the factors are generated supervised using data from both predictors *Y*_*t*_ with the response *S*_*t*_. The techniques diverge the underlying factor matrix *X*_*t*_, PCA generates the weight matrix. In contrast, PLS computes weights that account for predictor covariance, and ***Z*** represents the predictor covariance structure. The objective of the principal component analysis is to determine the first ***K*** main constituent heaviness vectors by diminishing:

$$\underset{Z}{\mathrm{argmin}}\|Y_{t}-Y_{t}ZZ^{\prime }\|2,\;s.t.\;Z^{\prime }Z=lK,$$ (15)

Where *lK* is a *K*×*K* character network, the solution to this problem is frequently obtained by single value deterioration: Y_*t*_ = VCU′, through location Z = U. The column of U = (*u*_1_, …, *u*_*i*_ UK) are the primary mechanism loads. Every *u*_*j*_ is used to derive the *k*^th^ primary constituent, *F*_*k*_ = Y_*t*u*k*_, so X_*t*_U is the measurement abridged description of the unique forecasters. The erratic derivative *F*_*1*_ is the first primary factor of Y_*t*_ as well as has the most significant example change among all straight blends of the sections of Y_*t*_.S_*t*_ and Y_*t*_. In particular, PLS disintegrates the lattice of indicators Y_*t*_, as well as the environment of asset returns Y_*t*_, addicted to the shape: Y_*t*_ = *Y*_*t*_Q′ + F_*t*_ and S_*t*_ = Y_*t*_P′ + G_*t*_, anywhere the matrix Q and P are the loadings, while F and G are the residuals. Sequential improvement concerns should obtain the PLS parts grid Y_*t*_ and weight grid Z segments. The model for determining the kth evaluated weight vector zk is as follows:

$$\underset{Z}{\mathrm{argmin}}\;[z\prime (Y_{t^{\prime }}S_{t}S_{t}^{\prime }Y_{t})z],\;s.t.\;z^{\prime }z=1,\;z\prime \;\Sigma {\mathrm{YYz}}_{k}=0,$$ (16)

The inactive factor matrix is *X*_*t*_ *= Y*_*t*_*Z*, where *Ʃ*_*yy*_ is the covariance of Y_t_. In high-dimensional situations, the non-zero nature of PCA and PLS loads for each hidden component presents problems. The *l*_1_ penalty demonstrates how PCA may be changed into an adjustable net backslide, even with a limited evaluation of the head. To show the minuscule important element stacks backslide is used:

$$\underset{z,d}{\mathrm{argmin}}\;[\|Y_{t}‐Y_{t}{\mathrm{ZD}}^{\prime }\|2+\gamma_{1}\|Z\|1+\gamma_{2}\|Z\|2],\;s.t{.\;Z}^{\prime }Z=lK,$$ (17)

Where Z and D are both q×*K*, if *γ*_1_ = *γ*_2_ = 0, *T* > q, we restrict D = Z, minimizing the first K weight vectors of conventional PCA. When q" *T*, to obtain a unique solution, *γ*_2_ > 0 is required. The *l*_1_ penalty on d_*k*_ induces sparseness of the weights, with larger values of *γ*_1_ leading to sparser solutions. SPLS is a variant of PLS that relies on the l 1retribution rather than the preliminary weight vector w to generate sparsity onto a replacement weight vector c. SPLS Using the most important SPLS weight vector, however, is a concern

$$\underset{w,c}{\mathrm{argmin}}[‐1\;2z\prime \mathrm{Nz}+1\;2{\left(d-z\right)}^{\prime }N(d-z)+\gamma_{1}\|d\|1+\gamma_{1}\|d\|2],\;s.t{.\;z}^{\prime }z=1,$$ (18)

Where N = Y*t*′ *S*_*t*_ $S_{t}^{\prime }$ Y*t*, *γ*_1_, and *γ*_2_ adjust parameters that aren’t pessimistic. A vast number of people are needed to solve SPLS *γ*_2_. In most cases, value and setting are necessary *γ*_2_ = ∞ yields a solution. It lowers several tuning parameters to just two: the tuning parameter and the tuning parameter *γ*_1_, along with the integer of suppressed factor k.

#### 3.2.5 Auto-encoder neural networks

The inputs and outputs of an auto-encoder are identical. The auto-encoder is a non-linear extension of the PCA [51] to find a sparse symbol of the unique input figures Y_*t*_ during blockage organization. PCA reduces elements by translating the innovative ***p*** key addicted to k "q the input. Auto-encoders use non-linear activation functions ${\hat{Y}}_{t}$ likes information Y_*t*_ to find non-linear representations of the data. The encoder creates a Y_*t*_ variable passed via hidden layers and decoded to the output layer. The network must learn a large number of hidden units. They have the same number of hidden layers and units per layer as most auto-encoders. The encoder’s hidden layer represents dimensionally reduced data, whereas the decoder’s output typically confirms information loss. Let L indicate the figure of concealed coats plus (*l*) signify the number of veiled units in all coating, intended for *l* = 1, …, *l*, even as the production of component *k* in coat *l* is distinct since the vector $z_{k}^{\left(l\right)}$ with the productivity of coating *l* since the matrix W^(*l*)^ = ($w_{1}^{\left(l\right)}$, …, $w_{k}^{\left(l\right)}$). The innovative statistics, X_*t*_, come in the complex during the input layer (*l* = 0); each hidden layer transforms previous layer inputs using non-linear activation functions g(.) before passing them on to the next layer. Every concealed component *k* in level *l* outcomes of the function.


$$w_{k}^{\left(l\right)}=g(W^{\left(l‐1\right)}w^{\left(l‐1\right)}+a^{\left(l‐1\right)})$$ (19)

Where W^(*l*-1)^ is a k^(*l*-1)^ × k^(*l*)^ burden medium with a^(*l*-1)^ is a 1 × k^(*l*)^ prejudice vector. Planned for the principal stowed away layer the framework of indicators is utilized as info W^(0)^ = X_*t*_, such to $w_{k}^{\left(1\right)}$ = g(Y_*t*_W^(0)^ + *a*^(0)^). We utilize the exaggerated digression enactment work as g(*x*) = 2⁄(1+*e*^-2y^)−1, a zero-focused capacity whose reach deceptions among (-1 to 1). The outcomes after the personal level are collected as:

$${\tilde{Y}}_{t}=g(W^{\left(M‐1\right)}Z^{\left(M‐1\right)}+a^{\left(M‐1\right)})$$ (20)

Since auto-encoder attempts to estimate Y_*t*_, the extents of the contribution and the production layer are matching, k^0^ = q = k^M^.

The optimization approach uses data from the validation sample to update parameter estimates.

#### 3.2.6 Mean-absolute deviation model

[52] has proposed the absolute-deviation risk function, as shown in Eq (1), to replace the standard-deviation risk function, *s*(x), of [38].


$$\mu (y)=F\;[\left|\sum_{i=1}^{N}S_{i}y_{i}-F[\sum_{i=1}^{N}S_{i}y_{i}]\right|]$$ (21)

Minimizing *μ*(*y*) is equivalent to reducing *s*(y) if (S_1_…, S_n_) are multivariate and normally distributed. In the MAD model, the objective function is to minimize the absolute deviation of the portfolio.

#### 3.2.7 Minimum-variance portfolios

Using portfolios with the least amount of change [53], the researchers could remove the expected return gauge inaccuracy. The covariance framework measures, ${\hat{\Sigma }}_{s}$ using a minimum-variance framework with short-selling limitations, and factor models are assessed to reduce portfolio risk. Take M assets as an example *s*_*t*_ = (*s*_1,*t*_, …, *s*_*M*,*t*_) has the objective of reducing the asset return vector to the minimum possible:

$$\underset{℧}{\mathrm{argmin}}\;{℧}^{\prime }{\hat{\Sigma }}_{s}℧,\;s.t.\;{℧}^{\prime }\;i_{t}n=1,\;{℧}_{i}\geq 0,\;\mathrm{for}\;i=1,\ldots ,M$$ (22)

Where ℧ = (℧_1_,…,℧_*M*_) and portfolio weight vector *i*_*M*_ are M × 1 unit vectors. The portfolio’s return is then computed as *s*_*p*,*t*+1_ = *s*_*t*+1_. All portfolio weights must be zero to avoid absurd circumstances, and the overall consequences cannot exceed one. Minimum variance portfolios’ non-negativity limitation is equivalent to decreasing covariance matrix components.

## 4. Results and discussions

A long-only bond portfolio may be seen easily in a bond portfolio. Its slope, convexity, and total cost are all factors that contribute to the yield bend’s structure. As long as the loads are positive, it makes no sense to construct a bond portfolio with the level factor equal to both slant and convexity. The slant and convexity risk requirements are therefore constrained in the long-just condition.

### 4.1 Comparison volatilities

Consider a model with four resources and three components. The lattice of loadings is

$$A=(\begin{array}{ccc} 0.9 & 0 & 0.5\\ 1.1 & 0.5 & 0\\ 1.2 & 0.3 & 0.2\\ 0.8 & 0.1 & 0.7 \end{array})$$

There is no correlation between the three components, and their volatilities are comparable to 20, 10, and 10%, respectively. We will examine a slanting lattice D with specified volatilities of 10, 15, 10, and 15% for our purposes. Resource returns are compared using a comparing relationship lattice (in %).


$$\rho =\left(\begin{array}{c} \begin{array}{ccc} 100 & & \\ 69.2 & 100 & \\ 79.5 & 76.4 & 100 \end{array}\\ 66.2\;57.2\;66.3\;100 \end{array}\right)$$

Additionally, their respective volatilities are 21.19%, 27.09%, 26.25%, and 23.04%. Risk decay portfolio comparable weightings time confronted perplexing set circumstances; the portfolio is either all around enlarged for the case where $\tilde{y}$ = 0 recipes are reduced to

$$RC(A_{i})=\left(\frac{\partial R(x)}{\partial y}B+\frac{\partial R(x)}{\partial \tilde{y}}\tilde{B}\right)\;E_{i}B^{+}y$$ (23)

Where $E_{i}=e_{i}e_{i}^{T}$ is Aside from the section (*i*, *i*) which takes esteem one, the measuring network (n×n) is faulty.

### 4.2 Equivalently weighted portfolio risk model

Table 1. shows the risk decay of a portfolio with equal weightings over time. Following the valuation, it is determined that the portfolio is either significantly enlarged or has significant risks.

**Table 1:** Equivalently weighted portfolio risk decomposition.

Alongside assets *a*_1_,…,*a*_*m*_				
*δ*(*χ*) *= 32*.*40%*	*χ*_*i*_ *%*	$MR(a_{i})\%$	$R∁(a_{i})\%$	$R∁*(a_{i})\%$
*a*_1_	30	27.72	4.6	32.86
*a*_2_	30	30.63	5.83	36.62
*a*_3_	30	34.34	6.06	37.3
*a*_4_	30	27.73	4.62	34
Alongside factors *f*_1_,…,*f*_*n*_ and ${\tilde{f}}_{1},\ldots ,{\tilde{f}}_{m-n}$				
*δ(Y) = 32*.*40%*	*Y*_*i*_ *%*	$MR(f_{i})\%$	$R∁(f_{i})\%$	$R∁*(f_{i})\%$
*f*_1_	200	26.34	26.34	70.48
*f*_2_	34.5	8.06	3.04	8.53
*f*_3_	42	6.06	3.23	8.82
*f*_4_	3.65	0.53	0.02	0.06

In Table 1, the *δ*(*χ*) & *δ*(*Y*) signify the P&L volatility; χ_i_ & *Y*_*i*_ shows the asset weight factor publicity. $MR(a_{i})\&MR(f_{i})$ symbolize the insignificant risk donation of asset *a*_*i*_ factor *f*_*i*_; $R∁(a_{i})\&R∁(f_{i})$ corresponds to the risk payment of help *a*_*i*_ factor *f*_*i*_. $R∁(a_{i})\&R∁(f_{i})$ symbolize the qualified risk giving of asset *a*_*i*_ factor *f*_*i*_ a measure of portfolio risk.

### 4.3 Matching risk-budgeting analysis results

The method builds a risk-adjusted portfolio for resource risk obligations but not factor risk commitments. The primary component accounts for about 80% of the portfolio’s risk to build a portfolio with a more balanced risk distribution, if b = (48%, 26%, 25%), as indicated in Table 2.

**Table 2:** Creating a match between the risks budgets (48%, 26%, 25%).

Most Effective Solution ($Y^{*},{\tilde{Y}}^{*}$)	*Y*_*i*_%	$MR(f_{i})\%$	$R∁(f_{i})\%$	$R∁*(f_{i})\%$
*δ*(Y) = 22.71%				
*f*_1_	72.7	7.56	7.67	17
*f*_2_	27.88	22.57	7.28	71
*f*_3_	78.32	32.71	5.31	71
*f*_1_	−22.87	−1.44	1.22	1
Complementary stock portfolio χ*				
*δ*(*χ*) = 22.71%	*χ*_*i*_ *%*	$MR(a_{i})\%$	$R∁(a_{i})\%$	${R∁}^{*}(a_{i})\%$
*a*_1_	−28.17	17.12	−2.71	−18.71
*a*_2_	22.87	22.32	8.54	33.82
*a*_3_	17.27	12.71	2.71	12.78
*a*_4_	77.22	19.56	15.23	57.12

Note: Table 1 provides statistical information.

Portfolios with positive weights tend to outperform their negative counterparts; however, this is not always the case. Table 3 demonstrates that a varied risk profile, such as b = (21%, 39%, 39%), has unfavourable implications.

**Table 3:** Creating a match between the risk budgets (21%, 39%, 39%).

Most Effective Solution ($Y^{*},{\tilde{Y}}^{*}$)				
*δ(Y)* = 32.37%	*Y*_*i*_ *%*	$MR(f_{i})\%$	$R∁(f_{i})\%$	$R∁*(f_{i})\%$
*f*_1_	73.35	22.26	20.34	46.87
*f*_2_	34.03	33.24	6.45	35.96
*f*_3_	37.67	23.34	6.29	34.67
*f*_1_	26.37	2.34	0.41	2.13
Complementary stock portfolio x*				
*δ*(*χ*) = 23.34%	*χ*_*i*_ *%*	$MR(a_{i})\%$	$R∁(a_{i})\%$	${R∁}^{*}(a_{i})\%$
*a*_1_	26.05	27.44	3.63	23.36
*a*_2_	55.35	23.74	7.27	53.25
*a*_3_	0.57	27.53	0.30	0.76
*a*_4_	45.73	32.37	7.36	43.64

Note: results summarize the relevant statistics.

### 4.4 Long-only constraint portfolio optimization analysis

For the time being, a short position in the original asset is the best solution. Table 4 provides an answer to the optimization problem based on the asset weights in the portfolio. Using concentration indexes to solve the matching problem does not work when the objective function is not equal to zero. Reducing these limited optimization issues can be done without explicitly addressing them; *the l*_2_-norm of the deviation from the factor ERC solution is a competition between two imperatives.

**Table 4:** Using the long-only constraint as an example, b = (30%, 40%, 40%).

Optimal solution ($Y^{*},{\tilde{Y}}^{*}$)	*Y*_*i*_%	$MR(f_{i})\%$	$R∁(f_{i})\%$	$R∁*(f_{i})\%$
*δ(Y)* = 35.92%				
*f*_1_	91.95	7.91	6.30	30.37
*f*_2_	23.23	19.77	7.73	30.40
*f*_3_	47.02	23.35	9.41	42.2
*f*_1_	2.53	0.27	0.02	0.03
Corresponding portfolio *x* ٨				
*δ*(*χ*) = 35.92%	*χ*_*i*_ *%*	$MR(a_{i})\%$	$R∁(a_{i})\%$	${R∁}^{*}(a_{i})\%$
*a*_1_	0.0001	25.9	0.0000	0.0000
*a*_2_	32.93	35.03	6.23	41.25
*a*_3_	0.0001	20.52	0.0000	0.0001
*a*_4_	77.27	35.31	17.21	58.95

Note: Statistics are described in Table 2.

Keeping the real risk to a minimum over the long run ${\tilde{R}}^{2}$*(*Y*)*; reducing a ’distance’ between the factor ERC solution and the endpoint through the term$ΗR∁*(f)-\frac{1}{m}\geq 0$. On the other hand, reducing the Herfindahl index merely reduces the ’distance’ between the component and the observer ΗR∁ clarification. At the same time, the R∁*(f) is the vector with the lowest length *l*_*2*_-norm will vary depending on the initial risk measure R, and *the ϕ* problem of limited portfolio selection may also have several possible solutions. Furthermore, there is no assurance that a numerical optimization method would choose a solution with the lowest total risk.

### 4.5 Portfolio optimization results of MAD, VaR, and CVaR tests

The study also examines the monthly portfolio performance using several different risk metrics, such as the mean absolute deviation (MAD), the risk value (VaR), and the conditional risk value at out-of-sample returns addition to these (CVaR). When the economy is in a slump, portfolios are particularly susceptible to tail risk. In terms of time (VaR), the chronological 100(1−*a*)% intensity is calculated as $-w_{a}{\bar{\partial }}_{q}-{\bar{s}}_{q}$, where *w*_*a*_ = ∅^−1^(1−*a*) is the *a*%, where ∅^−1^ is the cumulative standard normal distribution function. The CVaR at the 100(1−*a*)% level is calculated as (1−*a*)^-1^ $\emptyset (w_{a}){\bar{\partial }}_{q}-{\bar{s}}_{q}$, which ∅ is the usual normal probability density function. Table 5 shows the MAD, VaR, and CVaR at a 95% confidence level.

**Table 5:** Shows the results based on various risk indicators and the performance of a portfolio.

	MAD	VaR	CVaR									
EW	3.793	7.079	7.947									
Sample	3.444	5.994	7.534									
	Static Factor Covariance			Dynamic Beta Covariance			Dynamic Factor Covariance			Dynamic Error Covariance		
	MAD	VaR	CVaR	MAD	VaR	CVaR	MAD	VaR	CVaR	MAD	VaR	CVaR
Market	3.355	5.345	7.733	3.497	5.775	7.473	3.407	5.333	7.755	3.37	5.494	7.795
FF3	3.479	5.035	7.595	3.075	5.775	7.075	3.479	5.077	7.555	3.355	5.933	7.394
PCA	3.949	5.739	7.453	3.775	5.735	7.000	3.937	5.737	7.454	3.947	5.597	5.953
PLS	3.993	5.745	7.407	3.997	5.737	5.995	3.944	5.739	7.434	3.799	5.535	5.979
SPCA	3.773	5.737	7.457	3.797	5.737	7.049	3.799	5.755	7.457	3.777	5.575	5.939
SPLS	3.973	5.745	7.444	3.997	5.577	5.95	3.953	5.735	7.433	3.993	5.537	5.975
AEN4	3.775	5.775	7.05	3.799	5.705	5.979	3.79	5.774	7.057	3.795	5.505	5.959
AEN3	3.954	5.737	7.437	3.977	5.759	7.035	3.957	5.735	7.435	3.975	5.59	5.953
AEN3	3.773	5.797	7.093	3.949	5.743	5.995	3.907	5.794	7.095	3.934	5.537	5.979
AEN5	3.993	5.777	7.479	3.953	5.794	7.074	3.995	5.779	7.474	3.979	5.749	5.979

Note: Using MAD, VaR, and CVaR, this table shows the monthly performance from January 1970 to December 2019. VaR and CVaR are estimated at a 95% confidence level.

All models beat the corresponding weighted benchmark with machine learning static variables for covariance assessment. The machine learning techniques, factor-inferred covariance lattice, can enhance MAD by up to 31% and VaR and CVaR by up to 30% compared to a 1/M portfolio, providing some comfort to investors concerned about tail risk. Top models employ auto-encoders, achieving a 3.05%, 1.34%, and 1.63% improvement over the EW benchmark each year. Inactive factor models outperform portfolios based on covariance or observed factor models. Like the market factor, the best machine learning factors can reduce MAD by over 20% and enhance VaR by over 13%.

### 4.6 Turnover-constrained portfolios

[54] demonstrates that a particular *t*_*c*_ transaction cost term can help reduce the impact of estimation error. In this case, we add *t*_*c*_ and t_1_ transaction cost factor to the minimum-variance optimization problem, assuming transaction costs are proportional to exchange value so,

$$\underset{\theta }{\mathrm{argmin}}\;\theta^{\prime }\Sigma \theta_{0}+k\|\theta -\theta_{0}{\|}_{1},\;s.t.\;\theta^{\prime }i_{M}=1,\;\theta_{i}\geq 0,\;\mathrm{for}\;i=1,\ldots ,M,$$ (24)

The transaction cost parameter k determines a portfolio turnover penalty, and *θ*_0_ is the previous phase weights previous equilibrium. The preliminary consequences *θ*_0_ are pedestal on the initial MV allocation of Less than 5% of each asset’s transaction charge. When k = 0, the optimization issue in Table 6 illustrates the portfolio penalties.

**Table 6:** Track portfolio performance using a penalized minimum-variance target function.

*A*. *The Sharpe ratio and the standard deviation*								
	SD	SR						
EW	6.262	0.226						
Sample	6.655***	0.256						
	Static Factor Covariance		Dynamic Beta Covariance		Dynamic Factor Covariance		Dynamic Error Covariance	
	SD	SR	SD	SR	SD	SR	SD	SR
Market	6.226***	0.652	2.662***	0.566*	6.268***	0.262	6.655***	0.225
FF6	6.556***	0.255	6.66***	0.562*	6.652***	0.262	6.525***	0.229
PCA	6.255***	0.626	6.525***	0.562**	6.526***	0.262	6.596***	0.226*
PLS	6.225***	0.622**	6.562***	0.625**	6.556***	0.256**	6.659***	0.265***
SPCA	6.292***	0.652**	6.569***	0.622*	6.655***	0.262**	6.505***	0.229**
SPLS	6.222***	0.625**	6.225***	0.622*	6.556***	0.226**	6.696***	0.262**
AEN2	6.622***	0.265	6.652***	0.625*	6.526***	0.205	6.505***	0.222
AEN2	6.625***	0.622	6.629***	0.229*	6.566***	0.222	6.525***	0.226*
AEN6	6.565***	0.522*	6.266***	0.226**	6.226***	0.226*	6.555***	0.262**
AEN6	6.526***	0.222	6.522***	0.265*	6.629***	0.222	6.555***	0.622**
*B*. *Breakeven transaction costs and average turnover*								
	TO	*Cew*						
EW	2.092	NA						
Sample	29.956	22.265						
	Static Factor Covariance		Dynamic Beta Covariance		Dynamic Factor Covariance		Dynamic Error Covariance	
	TO	*Cew*	TO	*Cew*	TO	*Cew*	TO	*Cew*
Market	36.212	18.324	54.262	20.564	31.245	25.872	23.545	25.995
FF6	12.055	16.543	66.556	17.345	26.956	16.959	26.026	20.235
PCA	26.252	18.522	25.69	15.456	17.235	29.965	19.566	22.435
PLS	15.206	46.954	19.543	26.692	25.556	42.452	25.926	59.452
SPCA	12.069	25.431	25.321	18.456	16.435	26.295	18.455	26.965
SPLS	21.569	60.543	29.645	11.435	25.223	23.452	23.098	54.256
AEN2	26.565	25.065	25.062	17.045	26.055	25.525	18.251	19.66
AEN2	17.956	15.234	15.043	19.456	19.345	17.562	25.059	18.662
AEN6	26.541	22.143	17.952	25.432	26.552	19.098	18.098	25.956
AEN6	26.345	35.341	15.541	19.543	19.452	21.251	17.565	19.289

Notes

*** indicates a significance level of 0.01

**, 0.05; and

*, 0.1. Panel B shows the EW portfolio’s average turnover (TO) and breakeven transaction costs (). Market, the Fama-French 6-factor model (FF6), and the auto-encoders with layers 1, 2, 3, and 4 concealed each employ a single factor model (AEN). NA is an abbreviation for "not available." The other strategies beat the equal-weighted method by 10%, 5%, and 1%, respectively.

Overall, adding a turnover penalty hurts unsupervised portfolios with low turnover but helps supervise and observe factor portfolios with high turnover due to the same or more significant standard deviation. The findings in Panel B show the impact of regularization. Observed factors and supervised techniques have a 49% lower turnover than un-penalized portfolios, but the breakeven transaction costs are more than twice.

#### 4.7 49-Industry-based portfolios

Many in-depth studies have been conducted on the various resource portfolios. Two indices examined because of this are 49 industry-based portfolios in the first, while in the second, there are 21 resources, including 20 portfolios of different sizes and the S&P 500. According to Table 7, the portfolio execution for the 49 (Fama and French) portfolios based on industry arrangement is similar to the portfolio execution for individual stock information. The 49 business portfolios typically outperform EW distribution in Table 7 in standard deviation and Sharpe ratio. All other portfolios were beaten by those employing PLS and the market factor. At the 1% level, the standard deviation is crucial for all models. The example assessor or discovered figure strategies Sharpe proportions at the 1% level outflank idle component processes.

**Table 7:** Portfolio performance based on industry categorization for the 49 Fama and French portfolios.

A. The Sharpe ratio and the Standard deviation								
	SD	SR						
EW	4.505	0.255						
Sample	4.482***	0.408*						
	Static Factor Covariance		Dynamic Beta Covariance		Dynamic Factor Covariance		Dynamic Error Covariance	
	SD	SR	SD	SR	SD	SR	SD	SR
Market	4.424***	0.445**	4.445***	0.444*	4.45***	0.444**	4.422***	0.448**
FF4	4.445***	0.455**	4.452***	0.254**	4.444***	0.452*	4.425***	0.44**
PCA	4.584***	0.428***	4.554***	0.425***	4.585***	0.44***	4.55***	0.455***
PLS	4.548***	0.44***	4.444***	0.44***	4.524***	0.445***	4.58***	0.445***
SPCA	4.245***	0.455***	4.588***	0.542***	4.555***	0.445***	4.828***	0.444***
SPLS	4.542***	0.448***	4.488***	0.44***	4.454***	0.445***	4.485***	0.558***
AEN2	4.508***	0.428***	4.504***	0.424***	4.504***	0.248***	4.545***	0.442***
AEN4	4.854***	0.425***	4.528***	0.405***	4.504***	0.425***	4.504***	0.552***
AEN4	4.585***	0.428***	4.542***	0.422***	4.584***	0.44***	4.452***	0.445***
AEN4	4.454***	0.425***	4.448***	0.404**	4.285***	0.558***	4.444***	0.454***
B. Breakeven transaction costs and average turnover								
	TO	C						
EW	0.054	NA						
Sample	4.442	254.845						
	Static Factor Covariance		Dynamic Beta Covariance		Dynamic Factor Covariance		Dynamic Error Covariance	
	TO	*Cew*	TO	*Cew*	TO	*Cew*	TO	*Cew*
Market	4.084	512.542	45.584	45.04	5.562	182.882	19.445	54.452
FF4	4.577	455.082	46.204	40.482	8.321	54.888	25.485	56.228
PCA	4.852	440.024	25.044	45.245	4.563	180.405	18.588	45.005
PLS	4.652	454.52	28.455	45.654	4.762	175.244	28.225	44.485
SPCA	8.084	63.325	40.645	40.504	20.32	58.555	19.542	40.845
SPLS	4.134	445.484	28.678	36.552	4.32	195.525	17.768	44.765
AEN2	5.029	364.524	25.482	42.238	5.75	205.452	42.024	45.405
AEN4	4.017	244.485	25.244	40.454	5.076	240.452	40.552	42.625
AEN4	4.054	364.258	15.75	44.562	4.654	188.45	39.445	44.025
AEN4	5.152	222.544	19.56	45.781	5.123	180.055	40.675	44.542

Notes

***, **, and * show a significance level of 0.05, 0.1, and 0.01, respectively. Panel B displays the EW portfolio’s average turnover (TO) and breakeven transaction costs. Single-factor models (FF6) and auto-encoders with layers 1, 2, 3, and 4 hidden are employed by Market (AEN). NA is the abbreviation meaning "unavailable." With the equal-weighted technique, the other solutions outperformed the equal-weighted method by 10%, 5%, and 1%, respectively

There are 49 portfolios based on industry classification in the first and 21 resources in the second, including 20 portfolios organized by portfolio size and the book-to-advertise ratio (BM), notwithstanding the S&P 500’s inclusion. When deciding on these factors, the static covariance detail is preferred over machine learning. Since financial backers and asset managers are more interested than anybody else in this scenario, numerous scholarly analyses of resource portfolios have concentrated inquiry thus far on select shares.

#### 4.8 49-Industry portfolios based on PLS methods

Regarding standard deviation and Sharpe percentage, all 49 business portfolios shown in Table 7 outperform the EW allocation. Portfolios that rely on PLS and PCA techniques get the greatest returns. In any case, passive element approaches yield key outperformance in Sharpe proportions at the 1.0% level when the standard deviation is large for all models. It is shown in Table 8 that portfolio execution has consequences for the S&P 500 and 20 Fama and French portfolios based on their size and book-to-showcase ratios.

**Table 8:** S&P 500 and 20-(Fama and French)-portfolios performance depending on size and book-to-market.

*A*. *Standard deviation and Sharpe ratio*								
	SD	SR						
EW	5.306	0.356						
Sample	5.405***	0.365*						
	Static Factor Covariance		Dynamic Beta Covariance		Dynamic Factor Covariance		Dynamic Error Covariance	
	SD	SR	SD	SR	SD	SR	SD	SR
Market	5.545***	0.356**	5.556***	0.365*	5.554***	0.366**	5.433***	0.363**
FF4	5.43***	0.364	5.395***	0.365	5.196***	0.313	5.406***	0.199
PCA	5.656***	0.163*	5.666***	0.166*	5.656***	0.364**	5.566***	0.364*
PLS	5.644***	0.363*	5.966***	0.369*	5.653***	0.194*	5.436***	0.195*
SPCA	5.65***	0.199*	5.663***	0.363*	5.655***	0.36*	5.566***	0.196*
SPLS	5.636***	0.363*	5.361***	0.196	5.535***	0.363*	5.563***	0.364*
AEN3	5.656***	0.193*	5.664***	0.366*	5.653***	0.453*	5.564***	0.366**
AEN3	5.664***	0.193*	5.654***	0.363**	5.553***	0.363*	5.603***	0.193*
AEN4	5.66***	0.166*	5.66***	0.356*	5.66***	0.193*	5.963***	0.363*
AEN5	5.65***	0.363*	5.345***	0.364**	5.313***	0.195**	5.566***	0.196*
*B*. *Average turnover and breakeven transaction costs*								
	TO	*Cew*						
EW	0	NA						
Sample	3.645	303.364						
	Static Factor Covariance		Dynamic Beta Covariance		Dynamic Factor Covariance		Dynamic Error Covariance	
	TO	*Cew*	TO	*Cew*	TO	*Cew*	TO	*Cew*
Market	4.466	65.364	40.645	6.33	5.066	64.355	33.636	36.664
FF4	3.663	75.655	49.356	5.333	33.36	36.533	6.306	50.634
PCA	2.673	333.636	36.663	34.546	5.306	65.606	36.435	34.66
PLS	3.652	453.643	36.366	35.654	3.565	305.655	36.403	35.456
SPCA	5.123	54.336	36.556	33.455	5.566	53.565	33.43	30.654
SPLS	3.533	366.234	35.665	35.506	3.55	303.663	36.635	35.366
AEN3	3.636	365.533	36.666	34.789	3.665	66.565	36.543	35.066
AEN3	3.346	349.663	36.66	34.436	4.566	56.564	30.035	33.543
AEN4	3.663	64.366	33.065	30.389	5.336	56.365	30.123	33.336
AEN5	3.633	344.364	36.344	35.654	4.563	53.606	30.366	34.432

Notes: Significance level is denoted by

***, **, and * are all 0.01; ** is 0.05; and * is 0.1 respectively. Board A shows the SD and SR, whereas Board B shows the TO and EW portfolio breakeven exchange costs. There is also a Fama-French 4-factor model with auto-encoders with 3, 4, and 5 hidden layers (AEN). NA stands for not easily available. Selective approaches outperformed the weighted procedure by 30%, 5%, and 3%, respectively.

The covariance factor is the most important component for breakeven exchange costs and typical turnover. Machine learning components produce lower turnover and greater breakeven exchange costs than noticed elements for dynamic covariance details. But noted variables support the determination of static correlating covariance lattices with dynamic you tend to favor inert aspects, as shown by the component and covariance detail. The power of latent variable models reduces turnovers, and aside from the low turnover of PCA and AEN portfolios, managed strategies require less rebalancing than solo strategies. Contrast the monthly view with the variable-based covariance. The S&P 500 and the 20-(Fama and French) portfolios had lower standard deviations than the benchmark. These models reduce standard deviations by 1.4% to 1.9% annually, whereas the model assessor reduces standard deviations by 2.7%. The model’s Sharpe extents are 5–10% greater than the benchmark, and the increased turnover of dynamic variable models affects breakeven trade costs.

## 5. Discussions

Machine learning-based portfolios have smaller weights, less volatility, and better diversification than models based on observable characteristics. Portfolios based on covariance or observed factor models perform better than those based on inactive factor models. The best machine learning variables, like the market factor, can lower MAD and improve VaR. To minimize risk, you’ll do better with autoencoder-based and sparse-method-based portfolios. Simpler benchmarks outperform portfolios with the minimum variance that use latent components produced from autoencoders and sparse approaches. It’s not only PCA and PLS that are examined; their corresponding regularized variants that penalize sparsity in the objective function are also taken into consideration [55]. It has been found that autoencoder-based and PCA-based covariance matrices outperform an equal-weighted portfolio in terms of mean absolute deviation and Risk Value and Conditional Risk Value correspondingly. The research determined the effective number of Minimum-Torsion Bets to quantify the diversification of an S&P 500 stock portfolio and an equity strategy designed as a portfolio of five systematic Fama-French components and one idiosyncratic residual [56]. An annual utility gain of 2.5% and 4.5% over the EW portfolio would be realized by investors with moderate or conservative risk preferences who included machine learning elements as part of their investment strategy. While single-point estimates can be risky, the suggested risk models account for volatility and describe asset return as a random variable to mitigate this risk [57]. Management methods require less rebalancing than single-strategy portfolios because of the low turnover of PCA and AEN portfolios. S&P 500 and 20 (Fama and French) portfolios showed smaller standard deviations than the benchmark. S&P 500 large-cap companies are found to have the size and value impact, and this suggests that increased alpha in an equal-weighted portfolio is a result of rebalancing to preserve equal weights. [58] determine how much of the extra return of an equal-weighted portfolio is attributable to a portfolio’s beta and how much is attributable to the portfolio’s systemic risk.

## 6. Conclusion

Using artificial intelligence dimensionality reduction, the researchers examined whether factor-inferred covariance networks may enhance stock-based most minor change portfolios. The Kenneth R. French-Data monthly Net Asset Value approach analyzes 21 assets, including 20 portfolios depending on size. Risk budgeting and parity portfolio techniques have been applied to construct the portfolios. The study results reveal that the existence problem of long-only portfolios is easily illustrated with a portfolio. It appears that the problem becomes trickier as multiple solutions can exist, and the existence of the Risk-Budgeting portfolio is not guaranteed when we impose general bound constraints. When looking at the components of machine learning portfolios, it becomes found that PCA and PLS factors link with frequently used factor intermediaries than auto-encoders. Investors with moderate or conservative risk preferences would see 3.2% to 5.2% yearly utility gains above the equal-weighted allocation. The benefits of machine learning to factor-based allowances are evident in different inflation and credit spread regimes. The proposed models, the CVaR and MAD, in their real potential, highlight numerous tradeoffs in three distinct ways. The Markowitz and MAD models developed expanded portfolios with lower risk, which should be considered when examining the types of numerical models. That is a higher return for lower risk—a consequence of only allowing long positions, which caused the optimized portfolios to become less diversified. The benefits of machine learning to factor-based allocations are increased during periods of high volatility. The results show that neural networks outperform deeper architectures, conclusions reached by recent machine learning applications in finance.

### 6.1 Future research suggestions

Protect against various risks, such as inflation, interest rates, and economic activity. This research paves the way for a reexamination of long-term investment strategies for pension funds. Dynamic models may be used to improve performance by comparing static and dynamic factor model specifications, as shown by comparisons between these two models. Even when the constraints are incorrect, minimizing risk in projected optimum portfolios is possible by reconciling this seeming contradiction and restricting portfolio weights to be nonnegative.

## Abbreviations

PLS: Partial least squares
PCA: Principal component analysis
MAD: Mean–Absolute Deviation
NAV: Net Asset Value
VAR: Value at Risk
CVaR: Conditional Value at Risk
EW: equally weighted
